# Mechanism of *Cornus Officinalis* in Treating Diabetic Kidney Disease Based on Network Pharmacology

**DOI:** 10.1155/2022/1799106

**Published:** 2022-07-09

**Authors:** Yuqing Zhang, De Jin, Rongrong Zhou, Cunqing Yang, Yuehong Zhang, Fengmei Lian, Xiaolin Tong

**Affiliations:** ^1^Guang'anmen Hospital, China Academy of Chinese Medical Sciences, Beijing 100032, China; ^2^Hangzhou Traditional Chinese Medicine Hospital, Nephrology Department, Hangzhou, Zhejiang, China; ^3^Institute of Metabolic Diseases, Guang'anmen Hospital, China Academy of Chinese Medical Sciences, Beijing, China

## Abstract

Diabetic kidney disease (DKD), one of the most important diabetic complications, is a great clinical challenge. It still lacks proper therapeutic strategies without side effects due to the complex pathological mechanisms. *Cornus officinalis* (CO) is a common traditional Chinese medicine, which has been used in the treatment of DKD and takes beneficial effects in therapy. However, the mechanism of CO in treating DKD is not clear yet. In this study, network pharmacology was applied to illustrate the potential mechanism of CO and the interaction between targets of CO and targets of disease. First, the active ingredients of CO and related targets were screened from the online database. Second, the intersection network between CO and disease was constructed, and protein–protein interaction analysis was done. Third, GO and KEGG analysis were employed to figure out the key targets of CO. Finally, molecular docking was carried out in the software SYBYL to verify the effectiveness of the ingredients and targets selected. According to GO and KEGG analysis, drug metabolism-cytochrome P450, sphingolipid signaling pathway, HIF-1 signaling pathway, TGF-beta signaling pathway, cGMP-PKG signaling pathway, estrogen signaling pathway, and TNF signaling pathway were most closely related to the pathogenesis of DKD. Moreover, NOS3, TNF, ROCK1, PPARG, KDR, and HIF1A were identified as key targets in regulating the occurrence and development of the disease. This study provides evidence to elucidate the mechanism of CO comprehensively and systematically and lays the foundation for further research on CO.

## 1. Introduction

Diabetes mellitus (DM) is a common clinical disease characterized by hyperglycemia resulting from insulin secretion deficiency or insulin resistance [1]. According to the different pathological mechanisms, diabetes could be classified into type 1 diabetes mellitus (T1DM) and type 2 diabetes mellitus (T2DM), and the occurrence of the latter one is more frequent in clinical. Diabetic kidney disease (DKD) is one of the most important microvascular complications of DM, especially T2DM, characterized by glomerular hyperfiltration, progressive albuminuria, and declining GFR, and has become the main cause of the end-stage renal disease (ESRD) [2]. According to the global fact sheet on diabetes published by the International Diabetes Federation (IDF), 537 million adults worldwide have suffered from diabetes by the end of 2021, and the number is expected to reach 643 million by 2030, and 783 million by 2045 (https://www.diabetesatlas.org/en/resources/). This rapid growth has had a significant impact on the prevalence rate of DKD in developed countries and has brought heavy medical burden to the society [3]. Therefore, how to find an effective treatment for DKD is a great challenge for the medical community.

According to the recent guidelines on the DKD treatment, lifestyle measures are generally the first choice of intervention. The treatment of DKD mainly focused on the control of hyperglycemia, blood pressure, and blood lipids. However, many individuals still suffer from DKD progression for the lack of available effective treatment. Thus, further in-depth research on the pathophysiological mechanisms and more novel therapies are urgently required. It is now gradually recognized that the major pathological mechanisms, including kidney inflammation [4], tubulointerstitial fibrosis [5], and oxidative stress [6, 7] play important roles in the progression of DKD. Previous research has observed an increase in the level of TNF-*α* and IL-6 in diabetic patients with albuminuria [8] and many studies both in vivo and in vitro have been conducted to attenuate the inflammation of renal cells by targeting chemokines such as MCP-1 and inflammatory cytokines such as TNF, NLRP3 [9], IL6, and IL18. Similarly, many studies are focusing on targets of renal fibrosis, such as TGF-*β* [10], p38MAPK [11], and HIF-1*α* [12]. These results suggest that renal damage may be mitigated by targeting the mechanisms above. However, because of the complex pathogenesis, studies on a single target sometimes are not enough to provide effective therapies for DKD. Various ethnomedical systems have long used plants and their extracts as part of complementary treatment for diabetes and its complications [13–16]. Traditional Chinese medicine (TCM) could take effect on complicated disease systems and multiple targets while reducing side effects at the same time. The interaction between compounds of Chinese herb and DKD targets can be elucidated by network pharmacology.

*Cornus Officinalis* Sieb. Et Zucc. (CO) is a widely used traditional Chinese medicine involved in multiple pharmacological activities, such as renal protection, anti-inflammation, antioxidation, and antidiabetes activity [17]. Previous research has demonstrated that CO and its abstracts have beneficial effects on metabolic disorders of DKD, including inflammation, oxidative stress, hyperglycemia, and the formation of advanced glycation end-products (AGEs) [18–20]. However, the molecular mechanism of CO in treating diabetic nephropathy is not clear yet. Therefore, this study is about to screen the active ingredients of CO and collect related targets to elucidate the mechanism of CO interacting with DKD targets.

Network pharmacology is an emerging approach to drug analysis, which takes multitargets into account rather than a single target [21]. Such a comprehensive and systematic research method is consistent with a holistic view and treatment based on syndrome differentiation of TCM [22]. By means of network pharmacology, the complex pathways of “ingredient-protein/gene-disease” can be elucidated, and the pharmacological action and safety of TCMs can be determined conveniently [23].

In this paper, network pharmacology was applied to illustrate the action mechanism of CO in treating DKD and the interaction between targets of CO and disease. First, active ingredients and related targets were screened from the online database. Second, the intersection network between CO and disease was constructed, and protein–protein interaction analysis was done. Third, GO and KEGG analysis were employed to figure out the key targets of CO. Finally, molecular docking was carried out to verify the effectiveness of the ingredients and targets selected. The workflow was exhibited in Figure 1.

## 2. Materials and Methods

### 2.1. Screening of Active Compounds of CO

The compounds of CO were collected from the Traditional Chinese Medicine Systems Pharmacology Database and Analysis Platform (https://tcmspw.com/tcmsp.php) [24]. Then the key parameters of oral bioavailability (OB) and drug-likeness (DL) were taken into consideration to screen the active compounds of CO. OB is one of the most commonly used pharmacokinetic properties in drug screening, which evaluates the absorption percentage of oral drugs objectively [25]. DL is a concept proposed for drug discovery that measures the absorption, distribution, metabolism, excretion, and toxicity (ADMET) of the drug affected by its pharmacokinetics [26]. In this study, ingredients with OB ≥ 30% and DL ≥ 0.18 were selected as active ingredients.

### 2.2. Collection of Compound Targets and Disease Targets

Pubchem ID of filtrated compounds was obtained from TCMSP to find the corresponding Canonical SMILES from Pubchem (https://pubchem.ncbi.nlm.nih.gov/). Related targets of these ingredients were predicted by inputting Canonical SMILES to the Swiss Target Prediction database (https://www.swisstargetprediction.ch/) with a species of “Homo sapiens.” Targets with the probability of 0 were removed from the result.

The DKD targets were collected from the Therapeutic Target Database (https://db.idrblab.net/ttd/), Online Mendelian Inheritance in Man (https://www.omim.org/), DrugBank (https://www.drugbank.ca/), and Disgenet (https://www.disgenet.org/) with “diabetic nephropathy” and “diabetic kidney disease” as search strategies, then the duplicates of targets from the four databases were removed.

### 2.3. Construction of Intersection Network and Analysis of Protein–Protein Interaction

The drug targets and DKD-related targets were intersected to obtain a disease-drug target's network, which was presented in a Venn diagram. Subsequently, Cytoscape 3.7.2 was employed to construct the intersection network as well as a compound-target network of CO. Next, we inputted the disease–drug targets into the String database (https://string-db.org/) to generate a protein–protein interaction network, setting the organism as “Homo sapiens,” and the image was presented by Cytoscape 3.7.2. Finally, we used the tool “network analyzer” to make a topological analysis of disease–drug targets, and the results tables of which were exported to a file. Among the results of a topological analysis, four indexes including degree, betweenness centrality, closeness centrality, and average shortest path length were considered crucial evaluations of the importance of nodes. The number of degrees, betweenness centrality, and closeness centrality has a positive correlation with the importance of nodes, whereas the smaller the average shortest path length, the more vital the node is in the network.

### 2.4. Gene Ontology and KEGG Pathway Enrichment Analysis

A gene list of intersection targets was uploaded to David database (https://david.ncifcrf.gov/) for gene functional annotation. The results of enrichment analyses of biological process, cellular component, and molecular function were arranged according to “*P* value” respectively, and the top 10 were selected and merged to form an enrichment GO term diagram. In the same way, the results of the main signaling pathways were obtained by KEGG pathway enrichment analysis, and an enrichment dot bubble diagram was drawn.

### 2.5. Molecular Docking Verification

Ten significant targets commonly involved in treating DKD were selected, referring to different algorithms and references. The PDB formats of targets-related proteins were downloaded from the Protein Data Bank (PDB) database. At the same time, five ingredients were chosen according to the degree, and their molecular structures were obtained in the TCMSP database and then we prepared the proteins by extracting ligand substructures, removing water, and adding hydrogens. Finally, the prepared proteins and molecules were docked in SYBYL-X 2.1.1 software using a semiflexible docking mode to verify the interaction between ligands and receptors [27]. The total scores calculated by SYBYL reflected the binding affinity and strength of the molecules [28], which were presented in a heatmap.

## 3. Results

### 3.1. Active Ingredients and Related Targets

There were 17 active ingredients selected from the TCMSP database according to OB and DL, which were summarized in Table 1. Among them, gemin D has the highest oral bioavailability of 0.68, and lanosta-8, 24-dien-3-ol, 3-acetate has the highest drug-likeness of 0.82. 0 398 compound-related targets were predicted in the Swiss target database, and the ingredient-target network made by Cytoscape 3.7.2 software was shown in Figure 2. As is shown in Figure 2, the hexagon node represents the ingredient node, and the diamond node represents the related target. The higher the degree, the closer the node color is to red, and the size of the node from small to big corresponds to the degree from low to high. We found that mandenol, hydroxygenkwanin, and tetrahydroalstonine had the most targets, ranking the first three. In addition, 170 disease-related targets were collected from TTD, OMIM, Drugbank, and Disgenet databases, among which were 32 overlaps intersecting with CO targets as shown in a Venn diagram in Figure 3. The disease targets were represented by blue circles, and the drug targets were represented by green circles. The overlapping part concluded 32 genes, which were considered key targets in subsequent studies to form visual networks.

### 3.2. The Network of Disease-Drug Targets and Protein-Protein Interaction Analysis

The 32 overlapping targets and 14 corresponding ingredients were imported to Cytoscape 3.7.2 to obtain a visual network and topological analysis, the result of which was shown in Figure 4. The diamond node represents the compound, and the octagon node represents the target related to both DKD and CO. The size of the node positively corresponds to the degree calculated by the topological analysis, which also means the significance of the gene. Similarly, the darker the color of nodes, the more vital the genes are. The top three ingredients are cornudentanone, mandenol, and tetrahydroalstonine, and the most important targets of CO on DKD are CYP2C19, PPARG, and UGT2B7.

Shown in Figure 5 is the result of protein–protein interaction analysis obtained by importing the above targets into the String database. The sequence of nodes is ranked by degree. The larger and the brighter the node is, the higher the degree is, and the more crucial role the target plays in treating DKD. The top 10 targets ranked by degree were summarized in Table 2, and the indexes of average shortest path length, betweenness centrality, and closeness centrality were all listed along. It can be seen in Table 2 that NOS3, SERPINE1, PPARG, TNF, and KDR may interact with 13 other targets, AGTR1 may interact with 12 other targets, HIF1A, MMP9, and MMP2 may be related to 11 other targets and NOX4 may be related to 8 other targets. These ten targets were considered the focus of PPI analysis.

### 3.3. GO and KEGG Enrichment Analysis of Key Targets

Gene list was submitted to David database for gene annotation including biological process, cellular component, and molecular function analysis, and obtained 75, 10, and 24 entries, respectively, with *P* < 0.05. The top 10 GO terms of each result were listed together in Figure 6. The analyses demonstrated that both positive and negative regulation of biological processes (BP) were involved in the treatment of DKD, including positive regulation of protein kinase B signaling, angiogenesis, ERK1, and ERK2 cascade, glycolytic process and vascular smooth muscle cell proliferation, negative regulation of blood pressure, and other processes, such as xenobiotic metabolic process, glucose homeostasis, response to drug, and angiogenesis. There are also many cellular components (CC) that take effect in the network, including the plasma membrane, organelle membrane, organelle, endoplasmic reticulum membrane, and Golgi apparatus. In terms of molecular function (MF), the genes are mainly concerned with heme binding, drug binding, ATP binding, transmembrane receptor protein tyrosine kinase activity, and so on.

19 potential pathways were predicted by analyzing 32 overlapping targets using KEGG enrichment analysis. As shown in Figure 7, the horizontal axis represents fold enrichment, and the vertical axis represents the KEGG pathway. The size of the bubble indicates the gene count of the pathway, and the color reflects the number calculated by the formula “−log10 (*P* value).” Among these pathways were eight predominant pathways that play important roles in the development of DKD, including Type II diabetes mellitus, drug metabolism—cytochrome P450, sphingolipid, HIF-1, TGF-beta, cGMP-PKG, estrogen, and TNF signaling pathways (Table 3). These eight pathways were the main items discussed later.

### 3.4. Molecular Docking Verification

A total of 10 common targets and top 5 compounds ranked by degree were docked in SYBYL-X 2.1.1 software, and scores of various aspects were calculated. The total scores are considered the main indication of binding capacity between ligands and receptors. As shown in Figure 8, the sequence of targets ranked by average total scores are as follows: NOS3, CYP2C19, TNF, ROCK1, PPARG, KDR, UGT2B7, ABCB1, HIF1A, and SERPINE1. Among the five compounds, mandenol, ethyl linolenate, and cornudentanone received higher scores. It suggests that they have better binding affinity to active targets.

## 4. Discussion

*C. officinalis* (CO) is a commonly used traditional Chinese medicine with a sour and astringent taste, which has the effect of tonifying liver and kidney, and invigorating qi and blood. The clinical application showed that CO had beneficial influences on the process of diabetic kidney disease. It could control hyperglycemia and ameliorate renal damage to exert renoprotective function [18, 29]. Moreover, CO is considered nontoxic to humans with no obvious side effects. Only mild gastrointestinal dysfunction was clinically observed after long-term use of CO. Also, the toxicity of CO was rarely reported in pharmacological experiments. The abstracts of CO were reported to have an insecticidal effect and may cause mild congestion in rabbit gastric mucosa [30].

Although CO has been widely used in treating DKD in clinical and gained therapeutic effects, its mechanism is still unclear. In this study, active compounds and targets of CO were selected, and the interaction between drug and disease was analyzed to reveal the mechanism in the treatment of DKD. In the development of pharmaceuticals, herbal products have always played an important role [31, 32]. Therefore, by exploring effective components, targets, and multichannel signaling pathways of CO, we can improve the success rates of animal experiments and clinical trials and reduce drug development costs, leading to more effective drug development.

It is well established that the major pathological changes of DKD include tubular inflammation, oxidative stress, autophagy, and, in advanced stages, glomerulosclerosis, atrophy, and interstitial fibrosis. Our studies have shown that the compounds in CO have multiple anti-inflammatory, antioxidant, and antifibrosis properties, protecting cells from damage and thus exerting its renal protective effect. The top five compounds of CO ranked by degree named cornudentanone, mandenol, tetrahydroalstonine, hydroxygenkwanin, and ethyl linolenate. A recent study showed that hydroxygenkwanin (HGK) was involved in anti-inflammation activity by decreasing the secretion of iNOS, NO, TNF-*α*, and IL-6 in macrophages and T lymphocytes [33, 34]. It is also demonstrated that HGK could attenuate the expression and accumulation of epithelial-mesenchymal transition (EMT)-related proteins, thereby alleviating renal fibrosis [35]. Furthermore, HGK was found to induce cell apoptosis to exert anticancer effects, which had proved to be effective in cancers such as oral squamous cell carcinoma [36], liver cancer [37], and nonsmall cell lung cancer [38]. The existing studies on HGK are not enough to uncover its biological functions from all aspects, but its anticancer effect has been an emerging hot spot both in vitro and in vivo studies. Moreover, its positive regulation of inflammation, EMT, and cell apoptosis indicates that HGK may work through similar mechanisms in the treatment of DKD, and it corresponds to the main histopathological changes of DKD such as inflammation, renal fibrosis, and oxidative stress. Similarly, the anti-inflammatory activity of ethyl linolenate (EL) was observed in dextran sulfate sodium (DSS)-induced mice. A study has shown that EL suppressed the production of NO and iNOS and may inhibit the transduction of NF-*κ*B/p65 signaling pathway in macrophage cells [39]. Cornudentanone was reported to have cytotoxic properties against cancer cells in vitro such as MCF-7, NCI-H460, and SF-268 [40]. Similar cytotoxic effects against cancer cell lines were identified for tetrahydroalstonine [41]. Furthermore, tetrahydroalstonine showed antibacterial potential, especially in Gram-negative infections [42]. Experimental verifications of the mechanisms of these ingredients are still lacking. It means the therapeutic effects on diabetic kidney disease could be explored from various aspects above, and more studies are needed.

The disease-drug and PPI network showed the interaction among targets and revealed their significance. According to PPI analysis and references from the biomedical literature database, the following genes were regarded as key targets in treating DKD: NOS3, TNF, ROCK1, PPARG, KDR, and HIF-1*α*. NOS3, one of the isoforms of nitric oxide (NO), whose abnormalities lead to the onset and development of DKD both in animal models and in the human body [43]. There was robust evidence demonstrating that the deficiency of NOS3 contributed to severe albuminuria, hypertension, mesangial expansion, the thickness of the glomerular basement membrane, and even glomerulosclerosis in different mouse models [44–46]. In humans, NOS3 genetic polymorphisms are associated with the susceptibility of DKD and promoted the progression of it [47, 48]. These all suggested that NOS3 played an essential role in the pathogenesis of DKD. TNF-*α* is a pleiotropic cytokine that acts as a predictive biomarker of renal function in diabetic patients. An increase of TNF, along with its receptors (TNFRs), was observed in patients with DKD [49]. Moreover, TNF is involved in the early stage of renal pathological changes by stimulating Na absorption and promoting renal hypertrophy [50]. Administrations that decreased the level of TNF reduced the inflammation response and exerted renoprotective effects [51]. The study also found that ROCK1 was involved in the occurrence of albuminuria in the STZ-induced mouse model by regulating the expression of megalin/cubilinand and TGF-*β*1 [51]. ROCK1 knocked-out mice showed protection against the loss of megalin/cubilin and thus restored albumin endocytosis to alleviate albuminuria [52]. In addition, the deletion of ROCK1 inhibited TGF-*β*1 expression and attenuated endothelial-to-mesenchymal transition (EndMT), which was directly responsible for renal interstitial fibrosis [53]. PPARG was expressed in renal glomeruli and tubules and associated with inflammation, oxidative stress, and renal insulin resistance [54]. Agonists of PPARG showed a renoprotective effect, which indicated that PPAGR might represent a potential target in treating DKD. KDR, also called VEGFR2, is one of the receptors of vascular endothelial growth factor (VEGF) and is directly correlated with the expression of VEGF [55]. An increase of KDR was observed in the early stage of DKD but not in long-term DKD [56], and it contributed to the renal structure changes by promoting mesangial matrix accumulation and neovascularization [57]. HIF-1*α*, mainly expressed in tubular cells, mediates the adaptive response to hypoxia, thus reaching a balance in terms of oxygen consumption and supply [58]. Besides, HIF-1*α* is associated with activating fibrotic genes such as *α*-SMA and fibroblast-specific protein-1 (FSP-1), resulting in an EMT process and eventually leading to renal fibrosis [12, 59]. In summary, these key targets play pivotal roles in the pathogenesis of DKD mainly from aspects such as inflammation, insulin resistance, oxidative stress, and fibrosis, and through these targets, CO might regulate clinical symptoms, including albuminuria and hypertension. It scientifically elucidated the function of CO in a multitarget way, which corresponded with the holistic view of TCM.

In KEGG analysis, drug metabolism—cytochrome P450, sphingolipid signaling pathway, HIF-1 signaling pathway, TGF-beta signaling pathway, cGMP-PKG signaling pathway, estrogen signaling pathway, and TNF signaling pathway were most closely related to the pathogenesis of DKD. The drug metabolism-cytochrome P450 pathway exerts its biological effects mainly through its derivative products epoxyeicosatrienoic acids (EETs) [60] and hydroxyeicosatetraenoic acids (HETEs) [61]. A study found that inhibition of HETEs and EETs prevented hyperglycemia-induced changes, including increased expression of TGF-*β* and overproduction of reactive oxygen species (ROS) [62]. It indicated that inhibition of cytochrome P450 signaling pathway had positive influences on fibrosis and oxidative stress in the kidney, and thus ameliorated renal injury and albuminuria [63]. Sphingolipid signaling pathway, touching multiple aspects of cellular function and pathophysiology, whose importance has been increasingly realized and highlighted nowadays [64]. There was a potential link between sphingolipids, especially in the most studied form sphingosine 1-phosphate (S1P), and proliferation of renal cells [65], inflammation, and tubulointerstitial fibrosis in DKD [66]. The study provided evidence that suppression of sphingolipids by Rapamycin treatment significantly reduced cell apoptosis in STZ-induced DKD mice [67]. HIF-1 signaling pathway performs a bidirectional function in different stages of the disease [68]. In most cases, it acts as a renoprotective molecular ameliorating hypoxia-induced damage and restoring tissue injury [69]. However, in the late stage of diabetic kidney disease, HIF-1-induced chronic hypoxia, and tissue repair activated ECM-associated proteins and contributed to renal tubule interstitial fibrosis [70]. In addition, the HIF-1 pathway was involved in many other biological processes, from erythropoiesis, angiogenesis, and inflammation to vascular calcification and apoptosis [58]. In recent years, Roxadustat, a new drug inhibiting HIF-1, was developed to treat renal anemia [71]. Studies showed that Roxadustat treatment for renal anemia in patients with or without dialysis increased hemoglobin levels and improved iron metabolism [72, 73]. TGF-*β*, along with its downstream targets, has been long regarded as profibrotic cytokines that directly regulate fibrosis-related pathogenesis such as extracellular matrix (ECM) deposition and epithelial to mesenchymal transition (EMT) [74, 75]. In addition, the TGF-*β* signaling pathway also has anti-inflammation effects, which might work by activating NF-*κ*B signaling [76, 77]. Studies demonstrated that inhibition of the TGF-*β* pathway reduced ECM deposition and attenuated fibrogenesis [78], whereas upregulated proinflammatory factors thus aggravated the inflammatory response [76], indicating a diverse role of TGF-*β* in the development of DKD. It is widely accepted that cyclic guanosine 5monophosphate (cGMP) could be stimulated by NO and thus activates its downstream targets, especially cGMP-dependent protein kinase (PKG), to exert biological functions [79]. A study found that high glucose conditions promoted advanced glycation end-products (AGE) accumulation, thereby downregulated the expression of NO-dependent cGMP and inhibited the cGMP-PKG signaling pathway [80]. A possible link between NO-cGMP-PKG signaling and renal fibrosis was revealed by the observation that induction of NO-PKG markedly inhibited AGE-induced proliferation of fibroblasts and activation of another fibrosis-related signaling [81]. Estrogen signaling pathway has proved to be a beneficial regulator of DKD, which ameliorated proteinuria and decreased ECM accumulation [82]. Estrogen signaling also has a cross-talk with TGF-*β* pathway, reducing TGF-*β*-induced collagen IV production, ultimately limiting the progression of fibrosis [83]. Studies suggested a possible involvement of TNF pathway in renal inflammation [84] and oxidative stress [85]. TNF-*α* could induce and magnify the inflammatory progression by increasing the level of adhesion molecules [86] and plasma inflammatory cytokines [87]. Furthermore, inhibition of TNF-*α* decreased the excretion of urinary albumin, partially indicating the mitigation of insulin resistance [88]. Taken together, these pathways take effect in various aspects of DKD, providing multiple therapeutic directions in the treatment of disease.

The clinical application of TCM has a history of thousands of years. Due to the complex chemical composition and the characteristics of multitarget and multipathway, the pharmacological research of TCM is often confronted with unclear composition, vague mechanisms, and disconnection between research basis and clinical application [89]. However, network pharmacology emphasizes integrity, systematization, and interaction, which can be used to explain the pharmacodynamic substances of TCM and their mechanisms. Our study shows that in the treatment of DKD, the main active components of CO mainly target NOS3, TNF, ROCK1, and PPARG, and regulate signaling pathways including drug metabolism-Cytochrome P450, sphingolipid, HIF-1, and TGF-beta to exert anti-inflammatory, antioxidant stress, and antifibrosis effects. These pharmacological characteristics provide a theoretical basis for the new drug discovery and provide guidance and support for the clinical application of CO. However, these results need to be further verified by experiments.

## 5. Conclusions

Based on network pharmacology analysis, the mechanisms of CO in the treatment of DKD were systematically revealed in a multi-ingredient and multitarget way. A total of 32 overlapping targets between disease and drug were collected, which corresponded to 14 active ingredients selected by the parameters OB and DL. The top three ingredients are cornudentanone, mandenol, and tetrahydroalstonine, and the most important targets of CO on DKD are CYP2C19, PPARG, and UGT2B7. Then we explored the potential targets and pathways involved in treating DKD by GO and KEGG analysis, among which six key targets and seven pivotal pathways were discussed in detail. It indicated that NOS3, TNF, ROCK1, PPARG, KDR, and HIF1A were key targets by which CO regulated the pathogenesis of DKD. Cytochrome P450, sphingolipid, HIF-1, TGF-beta, cGMP-PKG, estrogen, and TNF signaling pathways were considered pivotal pathways that are directly related to DKD. Finally, 5 active components and 10 commonly used targets were docked to reveal the binding affinity between them. It showed that the targets of NOS3, CYP2C19, TNF, ROCK1, and PPARG, and the compounds of mandenol, ethyl linolenate, and cornudentanone have better binding affinity. In conclusion, this study provides evidence to elucidate the mechanism of CO in a comprehensive and systematic way using network pharmacology.

## Figures and Tables

**Figure 1:** The workflow of network pharmacology.

**Figure 2:** The ingredient-target network of CO.

**Figure 3:** Venn diagram of the disease-drug intersection.

**Figure 4:** The network of disease-drug targets.

**Figure 5:** The network of protein–protein interaction.

**Figure 6:** The top 10 GO analyses of BP, CO, and MF.

**Figure 7:** KEGG pathway enrichment analysis.

**Figure 8:** The molecular docking heatmap of key compounds and targets.

**Table 1:** 17 active ingredients of CO.

Number	Mol id	Ingredients	OB (%)	DL
1	MOL001494	Mandenol	42	0.19
2	MOL001495	Ethyl linolenate	46.1	0.2
3	MOL001771	Poriferast-5-en-3beta-ol	36.91	0.75
4	MOL002879	Diop	43.59	0.39
5	MOL002883	Ethyl oleate (NF)	32.4	0.19
6	MOL003137	Leucanthoside	32.12	0.78
7	MOL000358	Beta-sitosterol	36.91	0.75
8	MOL000359	Sitosterol	36.91	0.75
9	MOL000449	Stigmasterol	43.83	0.76
10	MOL005481	2,6,10,14,18-pentamethylicosa-2,6,10,14,18-pentaene	33.4	0.24
11	MOL005489	3,6-digalloylglucose	31.42	0.66
12	MOL005503	Cornudentanone	39.66	0.33
13	MOL005530	Hydroxygenkwanin	36.47	0.27
14	MOL008457	Tetrahydroalstonine	32.42	0.81
15	MOL000554	Gallic acid-3-O-(6′-O-galloyl)-glucoside	30.25	0.67
16	MOL005552	Gemin D	68.83	0.56
17	MOL005557	Lanosta-8,24-dien-3-ol, 3-acetate	44.3	0.82

**Table 2:** Top 10 targets ranked by degree.

Name	Average shortest path length	Betweenness centrality	Closeness centrality	Degree
NOS3	1.65517241	0.08566654	0.60416667	13
SERPINE1	1.72413793	0.05417328	0.58	13
PPARG	1.55172414	0.29547763	0.64444444	13
TNF	1.5862069	0.09751356	0.63043478	13
KDR	1.82758621	0.11988307	0.54716981	13
AGTR1	1.72413793	0.18242736	0.58	12
HIF1A	1.79310345	0.01358883	0.55769231	11
MMP9	1.79310345	0.01358883	0.55769231	11
MMP2	1.79310345	0.04492826	0.55769231	11
NOX4	2.03448276	0.00950426	0.49152542	8

**Table 3:** Main pathways involved in treating DKD.

Term	Pathway	Genes
hsa04930	Type II diabetes mellitus	INSR, PRKCE, TNF, GCK
hsa00982	Drug metabolism—cytochrome P450	CYP2C9, CYP2C19, UGT2B7
hsa04071	Sphingolipid signaling pathway	ROCK1, NOS3, PRKCE, TNF, MAP3K5
hsa04066	HIF-1 signaling pathway	NOS3, INSR, SERPINE1, HIF1A
hsa04350	TGF-beta signaling pathway	ROCK1, TNF, TGFBR1
hsa04022	cGMP-PKG signaling pathway	ROCK1, NOS3, INSR, PRKCE, AGTR1
hsa04915	Estrogen signaling pathway	NOS3, MMP2, MMP9
hsa04668	TNF signaling pathway	TNF, MMP9, MAP3K5

## Data Availability

The data used to support the findings of this study are included within the article.
